# Mutual regulation of MDM4 and TOP2A in cancer cell proliferation

**DOI:** 10.1002/1878-0261.12457

**Published:** 2019-02-04

**Authors:** Tao Liu, Hailong Zhang, Sha Yi, Lubing Gu, Muxiang Zhou

**Affiliations:** ^1^ Department of Pediatrics and Aflac Cancer and Blood Disorders Center Emory University School of Medicine Atlanta GA USA

**Keywords:** cancer cell proliferation, MDM4, p53, TOP2A

## Abstract

MDM4 and topoisomerase IIα (TOP2A) are overexpressed in various human cancers. MDM4 acts as an oncoprotein which promotes cancer progression by inhibiting tumor suppressor p53. As a DNA replication‐ and cell division‐regulating enzyme, TOP2A is the main target of many anticancer therapy regimens; however, the exact role of TOP2A in cancer remains elusive. Herein, we report that MDM4 and TOP2A bind to each other and are mutually upregulated at the post‐translational level, leading to TOP2A protein stabilization, inhibition of p53, and increased tumor‐cell proliferation. We demonstrate that the C‐terminal region (CTR) of TOP2A binds to a unique sequence (residues: 188–238) of MDM4, which contains an auto‐inhibitory segment regulating the MDM4‐p53 interaction. TOP2A binding in turn activates MDM4 for p53 binding, resulting in enhanced inhibition of p53 and cancer cell proliferation. Conversely, binding of the MDM4 sequence to the CTR of TOP2A stabilizes TOP2A protein, leading to increased TOP2A protein expression. These results reveal novel functions of MDM4 and TOP2A as well as their interactions in oncogenesis, suggesting that inhibition of the MDM4‐TOP2A interaction may represent a novel strategy in specifically and simultaneously targeting TOP2A and MDM4 for cancer treatment.

**Abbreviations**
ALL: acute lymphoblastic leukemia
CTR: C‐terminal region
ITC: isothermal titration calorimetry
kDNA: kinetoplast DNA
KO: knockout
MDM4: murine double minute 4
NTR: N‐terminal region
TOP2A: topoisomerase IIα

## 1 Introduction

Topoisomerase II (TOP2) is a nuclear protein required for DNA replication and cell division (Watt and Hickson, 1994). The primary role of TOP2 is to decatenate intertwined DNA during anaphase to allow chromosome segregation to occur prior to cell division. TOP2 has therefore become the primary cellular target for many of the most widely used and effective chemotherapeutic drugs including doxorubicin, etoposide, and mitoxantrone, even though the exact mechanism of cell growth inhibition and killing remains unclear (Pommier, 1993).

Topoisomerase II has two genetically distinct isoforms (TOP2A and TOP2B) that are differentially expressed and regulated in living cells. While TOP2B is expressed in quiescent cells in virtually all tissues throughout the cell cycle, TOP2A is typically expressed at high levels in rapidly proliferating and growing cells and its expression is cell cycle‐regulated, peaking in G2/M (Woessner *et al*., 1991). High levels of TOP2A expression are also detected in diverse human malignancies; these include adrenocortical, nasopharyngeal and gallbladder carcinomas, and cancers of the breast, ovary, oral, esophageal, lung, liver, colon, and leukemia (Depowski *et al*., 2000; Faggad *et al*., 2009; Jain *et al*., 2013; Lan *et al*., 2014; Meng *et al*., 2012; Mueller *et al*., 2004; Towatari *et al*., 1990; Washiro *et al*., 2008). TOP2A overexpression in these cancers is associated with aberrant cell proliferation, aneuploidy, an aggressive tumor phenotype, advanced disease stage, tumor recurrence, and decreased overall survival (Doussis‐Anagnostopoulou *et al*., 2008; Faggad *et al*., 2009; Jarvinen *et al*., 1996; Kalogeraki *et al*., 2005; Lan *et al*., 2014; Nakopoulou *et al*., 2000; Zhao *et al*., 2008).

Murine double minute 4 (MDM4), also known as MDMx, is amplified or overexpressed in various human cancers (Danovi *et al*., 2004; Han *et al*., 2007; Li *et al*., 2014; Liang *et al*., 2010; Riemenschneider *et al*., 1999; Wade *et al*., 2013). Thus, overexpression of MDM4 appears to favor cancer cell survival. MDM4 was initially described as an MDM2 homolog inhibiting p53 tumor suppression activity (Shvarts *et al*., 1997). However, it appears to inhibit p53 by different mechanisms from MDM2. Although the N‐terminal region (NTR) of both MDM2 and MDM4 bind similarly to p53 to inhibit p53‐mediated transactivation, the p53‐binding activity of MDM4 (but not MDM2) is inhibited by an intramolecular sequence, located in the central region of MDM4 (Bista *et al*., 2013; Chen *et al*., 2015). Additionally, the C‐terminal RING domain of MDM2 has E3‐ligase activity to induce p53 ubiquitination. In contrast, the MDM4 C‐terminal RING domain lacks this activity, although MDM4 can bind to the MDM2 RING domain to enhance its E3‐ligase activity (Shadfan *et al*., 2012; Wade *et al*., 2010).

In the present study, we report an additional mechanism by which MDM4 inhibits p53 via interaction with TOP2A. We demonstrate that MDM4 and TOP2A interacted and mutually regulated each other, forming a positive feedback loop that stabilized both proteins leading to increased expression. Overexpression of TOP2A by MDM4 increased DNA catalytic activity, whereas increased MDM4 activity by TOP2A resulted in enhanced inhibition of p53, which increased cancer cell proliferation.

## 2 Materials and methods

### 2.1 Cells

This study used ten acute lymphoblastic leukemia (ALL) cell lines (EU‐1, EU‐2, EU‐3, EU‐4, EU‐5, EU‐6, EU‐10, EU‐11, EU‐12, and SUP‐B13) and 13 neuroblastoma cell lines (SH‐EP1, SH‐SY5Y, SK‐N‐SH, SK‐N‐AS, SK‐N‐BE1, SK‐N‐BE2, NB‐1691, NB‐1643, IRM‐32, IRM‐5, LAN‐1, LA1‐55N, and LA1‐5S). All EU cell lines were established from children with ALL at Emory University. SUP‐B13 was obtained from Stephen D. Smith (University of Kansas Medical Center, Kansas City, KS, USA). We obtained all NB lines from H. Findley (Emory University). All cancer cell lines were authenticated and confirmed as identical to those published in prior publications (Gu *et al*., 2012; He *et al*., 2011; Peirce *et al*., 2011; Zhou *et al*., 1995). The 293T and H1299 cell lines purchased from the American Type Tissue Collection (Bethesda, MD, USA) were used for CRISPR/Cas9 genome editing and gene transfection assays.

### 2.2 Plasmid and transfection

We constructed plasmids for full‐length and various 5′ or 3′ deletions of MDM4 by PCR and cloned into the pCMV‐myc vector. Similarly, plasmids of TOP2A and three TOP2A fragments (1–431, 432–1193, and 1194–1531) were cloned into the pCMV‐HA vector. We also generated plasmids for the MDM4 fragments (188–300, 421–490) and the TOP2A C‐terminal region (CTR; 1194–1531) in the bacterial pGEX expression vector to produce proteins for isothermal titration calorimetry (ITC) assay as described below. The p53 expression plasmid was provided by B. Vogelstein (Johns Hopkins University School of Medicine). Transfection of plasmids was performed in 6‐well plates, using Lipofectamine™ 2000 reagents (Invitrogen, Waltham, MA, USA) according to the manufacturer's instructions.

### 2.3 CRISPR/Cas9‐mediated MDM4 gene disruption and RNA interference

The MDM4 CRISPR knockout (KO) plasmids consisting of human MDM4‐specific 20 nt guide RNA sequences derived from the gecko (v2) library were purchased from Santa Cruz (Cat.No.: sc‐417855, Dallas, TX, USA). MDM4 KO was carried out using CRISPR/Cas9, and stable clones were selected after about 1 month of culture. The siMDM4 (sc‐37448) and sip53 (sc‐29435) lentivectors were purchased from Santa Cruz. The siTOP2A lentivector (i025065b) was purchased from ABM (Richmond, BC, Canada). Cells were infected with siMDM4 or siTOP2A lentiviral plasmids following the manufacturer's manuals.

### 2.4 Immunoprecipitation and western blot assay

For immunoprecipitation (IP), we lysed cells in a buffer composed of 50 mm Tris, pH 7.6, 150 mm NaCl, 1% Nonidet P‐40, 10 mm sodium phosphate, 10 mm NaF, 1 mm sodium orthovanadate, 2 mm PMSF, 10 μg·mL^−1^ aprotinin, 10 μg·mL^−1^ leupeptin, and 10 μg·mL^−1^ pepstatin. After centrifugation, the clarified cell lysate was separated from the cell‐debris pellet and then incubated overnight at 4 °C with 15 μL Protein G plus/Protein A‐agarose and 1 μg of antibodies. For western blot, the resulting cell lysates or immunoprecipitates were resolved by SDS/PAGE. Protein bands were transferred to a nitrocellulose filter, probed with specific antibodies, and quantitated using a chemiluminescent detection system (Pierce, Waltham, MA, USA).

Antibodies used in this study include MDM4 (2D10F4) from LifeSpan BioSciences (Seattle, WA, USA); TOP2A (RB‐117‐PO) from NeoMarkers (Portsmouth, NH, USA); MDM2 (SMP14) and Ub (U5376) from Sigma (St. Louis, MI, USA); p53 (DO‐1), TOP2B (H‐286), GAPDH (SC‐47724), and Bcl‐2 (N‐19) from Santa Cruz (Dallas, TX, USA); PUMA (ab9346) and p21 (12D1) from Cell Signaling (Danvers, MA, USA); HA (12CA5) from Roche (Branford, CT, USA); Myc (631206) from Clontech (Mountain View, CA, USA). All antibodies were used according to the manufacturers’ instruction.

### 2.5 Cycloheximide (CHX) chase assay

Protein turnover was assessed by a standard protein‐synthesis‐inhibitor cycloheximide (CHX) chase assay. Briefly, cells were treated with 50 μg·mL^**−1**^ CHX for different times before lysis, in the presence or absence of reagents; these were then tested by western blot analysis to reveal concurrent expression levels of tested proteins.

### 2.6 RNA extraction and qRT‐PCR

Total RNA was extracted from cells using the RNeasy Mini Kit (Qiagen, Germantown, MD, USA). First‐strand cDNA synthesis was performed with a mixture of random monomers and oligo‐dT as primers. Amplification was performed with a 7500 Real‐Time PCR System (Applied Biosystems, Beverly, MA, USA), using the QuantiFast SYBR Green RT‐PCR kit (Qiagen), according to the manufacturer's instructions. All specific primers for amplification of specific genes, as well as the housekeeper gene GAPDH, were purchased from Qiagen.

### 2.7 Isothermal titration calorimetry assay

The expression and purification of GST‐fused MDM4 (188–300) and TOP2A CTR proteins were performed as described previously (Gu *et al*., 2009). For the ITC assay, 20 μm of TOP2A CTR protein was placed in a 400 μL buffer containing 10 mm HEPES at pH 7.2 and 150 mm NaCl, in a loading 96 DeepWell PP plate (Nunc; Thermo Fisher Scientific, Waltham, MA, USA). A 10‐fold concentration of MDM4 protein (200 μm) in 120 μL of the same buffer was automatically transferred by the auto‐ITC200 instrument (MicroCal, GE, Boston, MA, USA) into the sample cell. MDM4 solution (2 μL) was titrated stepwise into the TOP2A sample cell using a syringe, for a total of 16 injections (except that the first injection was 0.4 μL). The equilibrium time between two adjacent injections was 210 s. We determined the binding stoichiometry (*n*), binding constant (*K*_d_), and thermodynamic parameters (Δ*H* and Δ*S*) by fitting the titration curve to a one‐site binding mode, using origin software (Originlab Corporation, Northampton, MA, USA) provided by the manufacturer.

### 2.8 TOP2A catalytic activity assays

TOP2A catalytic activity was assayed by the decatenation of kinetoplast DNA (kDNA), using a TOP2 assay kit (TopoGEN, Port Orange, FL, USA), following manufacturer's instructions. Briefly, nuclear protein was extracted and incubated with 0.2 μg kDNA (Nippon Gene, Toiya‐machi, Toyama, Japan) in assay buffer (50 mm Tris/HCl, pH 8.0, 120 mm KCl, 10 mm MgCl_2_, 0.5 mm ATP, 0.5 mm DTT, and 30 μg·mL^**−1**^ BSA). After incubation for 10 min at 37 °C, reactions were stopped by the addition of stop buffer (5% sarkosyl, 0.0025% bromophenol blue, and 25% glycerol). The reaction products were analyzed on 1% agarose gels containing 0.5 μg·mL^**−1**^ ethidium bromide.

### 2.9 Cell proliferation and clonogenic assays

WST assay was used to measure cell proliferation. Briefly, an equal number of control or gene‐transfected cells were seeded in seven microtiter plates and cultured for 1–7 days. WST was applied for 4 h each day in consecutive plates before the OD was read.

A clonogenic assay to measure colony formation was used according to a previously described method (Franken *et al*., 2006). Briefly, cells were harvested with treatment by trypsinization, producing a single‐cell suspension, and then, 200 cells were seeded into a six‐well plate and cultured for ~ 2 weeks. Colonies were stained with a mixture of 6.0% glutaraldehyde and 0.5% crystal violet for 30 min. Then carefully removed the staining mixture, rinsed with tap water, and counted the colonies.

### 2.10 Flow cytometry

Flow cytometry was performed to analyze the cell cycle position. Cells were collected, rinsed twice with PBS, fixed in 70% ethanol for 1 h at 4 °C, washed twice in PBS, and re‐suspended in 0.5 mL PBS containing 20 μg·mL^**−1**^ of propidium iodide and 20 μg·mL^**−1**^ of RNase A. Following incubation at 4 °C for at least 30 min, the samples were analyzed using a FACScan (Becton Dickinson, Franklin Lakes, NJ, USA) with winlist software (Verity Software House, Inc., Topsham, ME, USA).

### 2.11 Statistical analysis

All data represent mean ± SD of three independent experiments. A two‐tailed *t*‐test was performed to compare the difference between two groups. A *P*‐value < 0.05 is considered significantly different, and *P *> 0.5 is considered not significant.

## 3 Results

### 3.1 MDM4 and TOP2A are concomitantly overexpressed and mutually regulated in cancer cells

Since overexpression of both MDM4 and TOP2A proteins contributes to cancer progression, we asked whether there is a link between MDM4 and TOP2A expression in cancer cells. We first performed western blot assays for MDM4 and TOP2A protein expression in 23 cancer cell lines, including 10 ALL and 13 neuroblastoma lines. We found that all cell lines expressed high levels of MDM4 and TOP2A, as compared with normal peripheral lymphocytes (NPL). A correlation of expression levels between MDM4 and TOP2A was noted in most lines (Fig. 1A, S1A,B); for example, EU‐4 and NB‐1643 overexpressed both MDM4 and TOP2A, whereas EU‐5 and LA1‐55N express relatively low levels of these proteins.

**Figure 1:** Expression and mutual regulation of MDM4 and TOP2A in cancer cells. (A) MDM4 and TOP2A protein expression in ALL and neuroblastoma cell lines was detected by western blot assays. (B) TOP2A expression in LA1‐55N cells transfected with MDM4 (tagged with myc) or control (vehicle) was detected by western blot, using anti‐myc antibody for indication of transfected MDM4. (C) Western blot for expression of TOP2A and MDM4 in NB‐1643 cells transfected with siTOP2A or control siRNA. (D) Western blot results show the expression of proteins as indicated in parental 293T cells (control) and 2 clones C19 and C28, in which MDM4 was silenced using the CRISPR/Cas9 (sgMDM4). (E) The expression levels of MDM4 and TOP2A mRNA relative to GAPDH in different 293T cells as in (D) were determined by quantitative RT‐PCR. Data represent mean ± SD of three independent experiments.

To further evaluate possible mutual regulation between MDM4 and TOP2A, we transiently transfected an MDM4 expression plasmid into LA1‐55N cells. Enforced overexpression of MDM4 resulted in increased expression of TOP2A (Fig. 1B). In contrast, siRNA‐mediated KO of TOP2A in NB‐1643 cells led to downregulation of MDM4 (Fig. 1C). Furthermore, we performed CRISPR/Cas9 genome editing to silence MDM4 (sgMDM4) in 293T and H1299 cell lines, yielding two MDM4‐null clones in 293T (Fig. 1D) and one in H1299 (Fig. S1C). As shown in these figures, the expression of TOP2A protein was also downregulated in MDM4‐null or MDM4‐reduced clones. Quantitative RT‐PCR demonstrated that the expression of TOP2A mRNA was not downregulated in the MDM4‐null clones of either the wt‐p53 293T (Fig. 1E) or the mutant‐p53 H1299 (Fig. S1D) lines (Higashitsuji *et al*., 2007; Yusein‐Myashkova *et al*., 2016), suggesting that MDM4 regulates TOP2A at the post‐transcriptional levels.

### 3.2 Interaction between MDM4 and TOP2A

We performed co‐IP and western blot assays using NB‐1643 cells to evaluate interaction between MDM4 and TOP2A. Results showed that MDM4 and TOP2A are mutually bound (Fig. 2A). In contrast, no binding activity was detected between either MDM2 and TOP2A or MDM4 and TOP2B.

**Figure 2:** MDM4 and TOP2A bind with each other. (A) co‐IP and western blot assays using antibodies as indicated for binding between endogenous MDM4 and TOP2A in NB‐1643 cells. WCE, whole cell extracts. (B) co‐IP and western blot for mapping the binding between transfected TOP2A CTR and different MDM4 fragments, using anti‐HA and anti‐myc antibodies, respectively. (C, D) ITC assays for binding of MDM4 (188–300) to TOP2A CTR (C) and no binding of MDM4 (421–490) and TOP2A CTR (D). The upper boxes show raw heating power over time, and the lower boxes are a fit of the integrated energy values, normalized for each injection.

Furthermore, we performed mapping studies to identify binding regions between MDM4 and TOP2A. Figure S2A showed the landmarks of TOP2A and MDM4 proteins. TOP2A contains three functional regions: (a) the NTR (1–431) with ATPase activity; (b) the central region (432–1193) involved in DNA interaction and cleaving; and (c) the CTR (1194–1531) involved in cell proliferation. MDM4 had an N‐terminal p53 binding region (19–102), central acidic and zinc‐finger regions (215–331), and a C‐terminal RING domain (437–483). In different from MDM2, MDM4 has a unique WWW motif (190–210), which inhibits interaction with p53.

We generated plasmids for various 5′ or 3′ deletions of MDM4 (1–420, 421–490, 1–200, 188–420, 188–300, 188–238, and 300–420) as well as for three functional regions of TOP2A. We first performed co‐transfection of MDM4 and TOP2A (full‐length and the three regions: 1–431, 432–1193, 1194–1531). Co‐IP and western blot assay results showed that MDM4 interacted with TOP2A CTR (1194–1531) and no binding activity was detected between MDM4 and the NTR or central region of TOP2A (Fig. S2B). Then, we performed co‐transfection of TOP2A CTR and various deletions of MDM4. Similar co‐IP and western blot demonstrated that the central region (188–420) of MDM4 bound to the CTR of TOP2A. As shown in Fig. 2B, MDM4 including either (1–420) or (188–420) bound to TOP2A CTR with the same affinity as full‐length MDM4. Binding was not detected between MDM4 NTR (1–200) and TOP2A CTR, or between MDM4 CTR (421–490) and TOP2A CTR. Further mapping found that the 50‐AA sequence (188–238) of MDM4 bound to TOP2A CTR.

We performed recombinant protein expression and purification assays for MDM4 (188–300) and TOP2A CTR (Fig. S2C) that were used for ITC analysis. Results confirmed that MDM4 (188–300) bound to TOP2A CTR with a binding *K*_d_ of 1.49 μm (Fig. 2C) and there was no binding between MDM4 CTR and TOP2A CTR (Fig. 2D). Additionally, in purification of the combination of MDM4 (188–300) and TOP2A CTR, we detected both proteins in a peak of gel filtration (Fig. S2D, peak 3 and lane 7), suggesting that recombinant MDM4 (188–300) and TOP2A are bound with each other to form heterodimers.

### 3.3 Mutual regulation of MDM4 and TOP2A at the post‐translational level

Since MDM4 and TOP2A bind at the protein level, we hypothesized that the correlated expression of these proteins occurs at the post‐translational level through protein modification. Thus, we performed CHX chase assay to test turnover of TOP2A in MDM4‐transfected cells. As seen in Fig. 3A, enforced overexpression of MDM4 increased the half‐life of TOP2A in LA1‐55N cells (expressing relatively low levels of MDM4 and TOP2A). In contrast, using siMDM4 to silence MDM4 in NB‐1643 cells (overexpressing MDM4 and TOP2A), we found that inhibition of MDM4 expression resulted in significant downregulation of TOP2A (Fig. 3B, lane 2). Furthermore, TOP2A downregulation was blocked by the protein degradation inhibitor MG132 (Fig. 3B, lane 4 vs lane 2), suggesting that MDM4 regulates TOP2A protein stability.

**Figure 3:** Mutual regulation of MDM4 and TOP2A through protein modification. (A) LA1‐55N cells were transfected with MDM4, and turnover of TOP2A in transfected cells was detected by CHX chase assay. Numerical labels under each TOP2A band represent their relative expression levels after normalization for GAPDH, as compared with untreated (0) samples that were defined as 1 unit. (B) NB‐1643 cells transfected with siMDM4 were treated with MG132 for 4 h and TOP2A expression detected by western blot. (C) CHX chase assay for MDM4 turnover in NB‐1643 transfected with siTOP2A. (D) Denaturing protein IP (using MDM4 antibody) and western blot (using ubiquitination antibody) for detection of MDM4 ubiquitination in siTOP2A‐ and control siRNA‐transfected NB‐1643 cells.

In addition, we performed similar CHX chase assays for MDM4 turnover in NB‐1643 cells transfected with siTOP2A. Inhibition of TOP2A resulted in rapid turnover of MDM4 (Fig. 3C). Further studies indicated that ubiquitination of MDM4 was increased in siTOP2A‐transfected NB‐1643 cells (Fig. 3D), suggesting that TOP2A regulates MDM4 protein stability through an ubiquitination mechanism.

### 3.4 Interaction between MDM4 and TOP2A increases TOP2A catalytic activity and MDM4‐mediated p53 inhibition

Since MDM4 stabilizes TOP2A protein, we evaluated whether the activity of TOP2A is increased due to enhanced expression of TOP2A in MDM4 overexpressing cells. The major function of TOP2A is DNA decatenation. We performed MDM4 gene transfection and measured its effect on TOP2A‐mediated decatenation of KDNA. In order to rule out the possible effect of p53 on TOP2A, we used the p53‐null cell line LA1‐55N (Gu *et al*., 2009). Results showed that enforced overexpression of MDM4 increased the decatenation of KDNA (Fig. 4A).

**Figure 4:** Effect of the interaction between MDM4 and TOP2A on TOP2A catalytic activity and p53 activation. (A) LA1‐55N cells were transfected with MDM4 and TOP2A catalytic activity detected by decatenation assay. (B) LA1‐55N cells co‐transfected with p53 and plasmids containing MDM4 DNA regions corresponding to either nucleotides 1–420 or 1–200 (tagged with myc), in the presence or absence of TOP2A CTR (tagged with HA). Transfected cells were immunoprecipitated with anti‐myc antibody. The expression of p53 and TOP2A CTR (HA) in the precipitates, and expression of p53 and TOP2A as well as MDM4 (myc) in whole cell extracts (WCE), was detected by western blot. (C) NB‐1643 cells were transfected with siTOP2A in the presence and absence of TOP2A CTR for the indicated times; protein expression was detected by western blot assay. (D, E) NB‐1643 cells were transfected either with siTOP2A alone (D) or with combination of siTOP2A and sip53 (D) for the indicated time, and cell cycle distribution was detected by flow cytometry. Data represent mean of three independent experiments, bars ± SD.

We performed co‐IP and western blot assays in LA1‐55N cells co‐transfected with p53 and either MDM4 (1–200) containing the p53‐binding sequence alone or MDM4 (1–420) containing binding sequences for both p53 and TOP2A, in the presence or absence of TOP2A CTR. Results showed that TOP2A CTR increased the binding between MDM4 (1–420) and p53 (Fig. 4B, lane 2 vs lane 1 of p53 IP panel), but not the binding between MDM4 (1–200) and p53 (lane 4 vs lane 3). However, the latter showed increased baseline binding (lane 3 vs lane 1) due to lack of the MDM4 auto‐inhibitory element.

Results as shown in Fig. 3C,D indicate that KO of endogenous TOP2A by siRNA results in MDM4 ubiquitination and protein degradation. To further evaluate whether TOP2A KO leads to activation of p53, we performed similar siTOP2A transfection in NB‐1643 cells and measured activation of p53 and its downstream targets p21 and PUMA. Inhibition of TOP2A resulted in increased expression of p53 as well as p21 and PUMA (Fig. 4C, right). This p53 activation was inhibited in the endogenous TOP2A KO cells co‐transfected with TOP2A CTR plasmid (Fig. 4C, left). Consistent with increased p53 and p21 protein expression, there was G1 cell cycle arrest in siTOP2A‐transfected NB‐1643 cells (Fig. 4D). In contrast, G1 cell cycle arrest did not occur in siTOP2A‐transfected NB‐1643 cells in the presence of sip53 (Fig. 4E).

### 3.5 TOP2A CTR promotes MDM4‐mediated cell proliferation and growth

We next evaluated the effect of TOP2A CTR‐mediated MDM4‐p53 binding and p53 activity on cancer cell proliferation. We first performed proliferation assays with SK‐N‐SH cells transfected either with TOP2A CTR and MDM4 alone or in combination. We selected the neuroblastoma cell line SK‐N‐SH for this study, because it expresses relatively low levels of TOP2A and MDM4 (Fig. 1A) and has a wt‐p53 phenotype (He *et al*., 2011). WST results showed that TOP2A CTR significantly stimulated cell proliferation when co‐transfected with MDM4, while TOP2A CTR transfection alone did not stimulate cell proliferation; similarly, MDM4 transfection alone only moderately increased proliferation (Fig. 5A).

**Figure 5:** Effect of TOP2A CTR on MDM4‐mediated cell proliferation and growth. (A) WST proliferation assay comparing the growth of SK‐N‐SH cells transfected with plasmids as indicated. *P <* *0.01. (B) colony assays of SK‐N‐SH and LA1‐55N cells transfected with plasmids as indicated, *P <* *0.01, as determined by two‐tailed *t*‐test. (C) representative colony formation of transfected SK‐N‐SK cells as in (B). (D) WST proliferation assay comparing the growth of different 293T cells (parental and sgMDM4 clones), *P <* *0.01. Data in (A, B, and D) represent mean ± SD of three independent experiments.

We also performed clonogenic assays for cell growth rate in SK‐N‐SH cells similarly transfected with the above plasmids. Consistent with WST assay results, TOP2A significantly stimulated colony formation when co‐transfected with MDM4, as compared with transfection of MDM4 alone (Fig. 5B,C). Additionally, we performed similar co‐transfections of TOP2A CTR and MDM4 in p53‐deficient LA1‐55N cells. We found no significant differences in colony formation among the cells with these different transfections (Fig. 5B). Because TOP2A CTR does not have ATPase and DNA‐regulation activity, we hypothesize that the TOP2A CTR proliferation‐enhancing activity in wild‐type p53 cells results from inhibition of p53 due to increased binding of MDM4.

Furthermore, we tested cell proliferation of 293T cells with MDM4 KO by CRISPR/Cas9, as compared with parental cells. Results showed that cell proliferation was significantly slower in sgMDM4 cells than in parental 293T cells (Fig. 5D). Since the expression of TOP2A was also downregulated in sgMDM4 cells, we believe the interaction between MDM4 and TOP2A is critical for cell proliferation and growth.

## 4 Discussion

To date, the primary role reported for MDM4 in oncogenesis is inhibition of tumor suppressor p53 either alone or via cooperation with MDM2. In the present study, we report an additional mechanism by which MDM4 inhibits p53 via interaction with TOP2A, resulting in cancer progression. Furthermore, interaction between MDM4 and TOP2A results in increased expression of TOP2A, which may also contribute to oncogenesis.

Murine double minute 4 protein consists of 490 amino acids with an N‐terminal p53 binding region, central acidic and zinc‐finger regions, and a carboxyl‐terminal RING domain. Although both MDM2 and MDM4 bind to p53 similarly through a hydrophobic pocket at their NTRs, the p53‐inhibiting activity of MDM4 (but not MDM2) is in turn inhibited by an MDM4 auto‐inhibitory sequence, located in the central region of MDM4 (Bista *et al*., 2013; Chen *et al*., 2015). Previous studies showed that casein kinase‐1 alpha (CK1α) binds to the central region of MDM4 and stimulates MDM4‐p53 binding (Chen *et al*., 2005; Wu *et al*., 2012). We found that TOP2A also binds to the central region of MDM4. We demonstrate that the CTR of TOP2A binds to the (188–238) region of MDM4, which contains the auto‐inhibitory sequence WWW (190–210) regulating MDM4‐p53 interaction (Bista *et al*., 2013). Consistent with the effect of binding by CK1α, TOP2A binding to MDM4 in turn stimulates MDM4‐p53 binding. We have further shown that increased binding of MDM4 and p53 mediated by TOP2A results in increased inhibition of p53 and cancer progression.

In addition, our results reveal a new function of MDM4: Binding of MDM4 to the CTR of TOP2A increased TOP2A protein expression. The expression of TOP2A is regulated by multiple mechanisms and multi‐step process with many potential points of control. For example, the TOP2A mRNA expression is associated with changes in proliferation state and cell cycle stage with high levels in rapidly proliferating cells and peaking in G2/M (Isaacs *et al*., 1998; Woessner *et al*., 1991). Additionally, the expression of TOP2A mRNA is negatively regulated by p53 (Sandri *et al*., 1996; Wang *et al*., 1997). Because MDM4 is an inhibitor of p53, overexpression of MDM4 could be able to increase TOP2A mRNA expression through inhibition of p53 and increased cell proliferation. In the present study, we demonstrated an additional mechanism for MDM4 to enhance TOP2A expression by stabilizing TOP2A protein.

Previous studies have demonstrated that MDM4 promotes genomic instability independently of MDM2 and p53 (Carrillo *et al*., 2015; Matijasevic *et al*., 2008a,b); however, its function in genome instability was unclear. Since TOP2A is a regulator of genomic instability, we speculate that the role of MDM4 in genomic instability is likely through regulation of TOP2A. It is known that the homeostatic balance of TOP2A in a normal DNA‐decatenating activity is critical for genomic stability and too few or too much of this protein will lead to topological stress on the chromosomes and chromosomal instability (Farr *et al*., 2014). Many previous studies have demonstrated that lack or too few of TOP2A causes chromosomal instability as chromosomes cannot be decatenated at anaphase (Carpenter and Porter, 2004; Dykhuizen *et al*., 2013; Johnson *et al*., 2009). The mechanism for abundant or too much TOP2A to confer chromosomal or other types of genomic instability is obscure. Although we demonstrate that the interaction between MDM4 and TOP2A increased TOP2A expression, the hypothesis that MDM4‐mediated genomic instability is through regulation of TOP2A needs to approve by further investigation.

Our results show that the interaction between MDM4 and TOP2A through binding of the central region of MDM4 and the CTR of TOP2A upregulates expression of both proteins. We have further demonstrated that this upregulation is due to protein stabilization. The mechanisms by which MDM4 stabilizes TOP2A and vice versa are not clear, although we have detected an increased ubiquitination of MDM4 in TOP2A‐null cells, suggesting that TOP2A has a de‐ubiquitination effect on MDM4. Since TOP2A has not previously been reported as a deubiquitinase, further study needs to be done to characterize this activity. Similarly, MDM4 may also stabilize TOP2A indirectly through regulation of ubiquitination activity. For instance, the tumor suppressor BRCA1 is a well‐characterized E3 ligase that regulates TOP2A ubiquitination and protein stabilization (Lou *et al*., 2005). Whether MDM4 interferes with BRCA1‐mediated TOP2A ubiquitination also needs to be investigated.

## 5 Conclusions

Possibly due to the auto‐inhibition of MDM4‐p53 binding, targeting of MDM4‐p53 interaction using small molecules has been unsuccessful, whereas several potent MDM2‐p53 inhibitors have entered clinical trials (Zhang *et al*., 2014). Because TOP2A CTR can increase MDM4‐p53 binding through interacting with the auto‐inhibitory element, targeting the interaction between TOP2A CTR and MDM4 auto‐inhibitory element may represent an alternative strategy to activate p53 in cancer cells by modulating MDM4 activity; simultaneously, targeting this interaction may result in specific downregulation of TOP2A. Chemotherapeutic drugs such as doxorubicin, etoposide, and mitoxantrone all have severe side effects, which is likely due to inhibition of TOP2B in normal cells, since these drugs target TOP2B as well as TOP2A (Lyu *et al*., 2007; McClendon and Osheroff, 2007; Zucchi and Danesi, 2003). Specifically inhibiting TOP2A by targeting the MDM4‐TOP2A interaction may represent an innovative approach for developing more effective and less toxic anticancer therapy.

## Conflict of interest

The authors declare no conflict of interest.

## Author contributions

MZ and LG conceived the project, designed the experiments and wrote the manuscript. TL, HZ and SY performed the experiments, analyzed, interpreted, and prepared data for publication.

## Supporting information


**Fig. S1.** Expression of MDM4 is associated with TOP2A protein expression in cancer cells.
**Fig. S2.** The CTR of TOP2A interacts to a unique sequence (188–238) of MDM4.
